# Design and Optimization of Aesthetic Education Teaching Information Platform Based on Big Data Analysis

This article has been retracted.

**DOI:** 10.1155/2022/5109638

**Published:** 2022-08-11

**Authors:** Xingxing Wu, Hai Gu

**Affiliations:** ^1^School of Finance, Jiangxi Institute of Economic Administrators, Nanchang 330088, China; ^2^School of Art, Mokwon University, Daejeon 35349, Republic of Korea; ^3^Department of IT Engineering, Mokwon University, Daejeon 35349, Republic of Korea

## Abstract

In the process of promoting school aesthetic education, some schools have some problems, such as insufficient construction of campus aesthetic education environment, lack of aesthetic thinking in various disciplines, and so on. In view of these problems, combined with the concept of the flipped classroom and the characteristics of artificial intelligence task-driven teaching, taking PHP, HTML + CSS + JS, and other development technologies as the main development technologies, and relying on the flipped classroom teaching mode of network learning space, this paper constructs an artificial intelligence core course website as a teaching platform for graduate teaching and undergraduate extended learning. The platform seeks the optimal solution of multiple combination optimization based on a genetic algorithm effectively improves the teaching quality of artificial intelligence courses and students' learning efficiency.

## 1. Introduction

Aesthetic education enhances aesthetic qualities, cultivates sentiment, warms the soul, stimulates innovation and creativity, and is an indispensable element in the overall development of students [1].

Aesthetic education informatization refers to the process of teachers incorporating modern information technology in the top-level system design, campus culture enhancement, teacher training, teaching platform construction, resource development, and implementation of teaching activities to accelerate the modernization of aesthetic education [2–4].

This document clarifies the why, what, and how of school aesthetic education in the new era, strengthening the nurturing function of school aesthetic education, which is an important model for guiding the whole society to value aesthetic education and creating a social atmosphere that jointly promotes the development of school aesthetic education [5]. Teachers should attach importance to aesthetic education and make it permeate and permeate all aspects of education and teaching. Information technology is a booster for improving the quality of education, and promoting aesthetic education with information technology is the direction and trend of education development and a necessary stage of education modernization [6]. At present, information technology in aesthetic education has become a new area of research in the field of aesthetic education, and its research is on the rise [7].

Aesthetic education is an important part of school education, and the construction of the campus environment is very important for cultivating students' aesthetic thinking. The campus environment can be a visual representation of a school's understanding and interpretation of aesthetic education [8]. However, some primary and secondary schools have a single style of campus environment construction and do not pay attention to the importance of the campus environment to the cultivation of students' aesthetic thinking, lacking an environmental design that reflects the unique local humanities, beautification style, and the core concept of campus culture [9].

The most pressing need in aesthetic education is the issue of teacher development. Nationally, there is still a considerable shortage of teachers for aesthetic education in terms of quantity, and even more so in terms of quality. [10] Interviews with some teachers and students revealed that there is a serious shortage of teachers with an arts background in some schools, so schools are lowering the bar when recruiting, which in turn leads to overall low quality of art teachers. In terms of curriculum arrangement, art and music courses are often taken up or switched at will by the main teachers, which leads to a lack of assurance in terms of class time and teaching quality in the Aesthetic Education curriculum [11].

Our schools have not invested enough in the infrastructure and teaching resources for Aesthetic Education's information-based teaching activities, and there is a general problem of low popularity and small scale. Although teaching resources in the information age have been greatly enhanced in terms of quantity, quality, and content, some teachers fail to select appropriate resources to make them fit with classroom teaching content when making use of the abundant teaching resources. At the same time, the construction of regional educational resource banks is in its infancy, and the use of information resources for the teaching of Aesthetic Education in Chinese primary schools is still far from the goal of abundant and effective use of resources [12].

Artificial Intelligence is a core course in the discipline of computer application technology. Through the study and practical application of this course, students can be trained to master the basic theories, cutting-edge technologies, and the ability to do things on their own and to be innovative [13]. Students are required to have a basic understanding of the classical algorithms and reasoning mechanisms of artificial intelligence theory and to develop intelligent systems based on the main research content after completing the basic theory and experimental teaching courses [14]. This requires a wide range of knowledge, deep basic theories, and strong practical skills in the teaching of AI courses [15–17].

In this paper, relying on the flipped classroom teaching mode of the online learning space, combined with the actual teaching cases based on the task-driven teaching mode, a website of artificial intelligence core courses is constructed as a teaching platform for postgraduate teaching and undergraduate extended learning, which effectively improves the artificial intelligence courses. Teaching quality and student learning efficiency.

## 2. Artificial Intelligence Web-Based Teaching Platform Positioning and Related Technologies

### 2.1. Online Teaching Platform Positioning

The construction of an online teaching platform for core courses in artificial intelligence mainly includes a flipped teaching concept, course content based on a task-driven teaching model, and an interactive and shared online platform. These two are complementary and mutually reinforcing. Secondly, mature network technology is needed to build the platform framework, so that the best course content can be displayed on the network platform, thus realizing the purpose of sharing and applying course resources [18]. In this paper, the teaching cases of AI core course teams in the past ten years are collected and collated, and an online teaching platform based on the flipped classroom teaching model is constructed.

### 2.2. Web-Based Teaching Platform Related Technologies

PHP is a server-side scripting language; MySQL is the most widely used Web database today. PHP and MySQL are a natural pair, and the combination of the two can be used to achieve many powerful features in web development. CSS makes it easy to control the appearance of a website's interface, making it easy to create web pages. CSS is also a great solution to the problem of page layout, making web pages smaller and faster to download [20].

## 3. Introduction to Traditional Genetic Algorithms and Hierarchical Decision Model

Genetic algorithms, or GA for short, are computational models that combine biological evolution and genetics. They can mathematically model the natural evolutionary process of organisms, corresponding the process of problem solving to the selection, crossover, and mutation of chromosomal genes during biological evolution and are thus used to find the optimal solution for multi-combination optimization.

The specific flow chart of the traditional genetic algorithm is shown in Figure 1.

The algorithmic components of a traditional genetic algorithm (GA) include chromosome encoding (containing the initialized population), fitness functions, and genetic operators (selection, crossover, variation). The traditional genetic algorithm firstly encodes and randomly generates an initial population, then conducts individual evaluation, and selection, determines whether to output, followed by random crossover and mutation operations and finally turns to individual evaluation to start a new cycle.

In order to establish a systematic risk assessment system for sports injuries, it is necessary to decompose the decision object based on the idea of the decomposition method and build a hierarchical model accordingly. According to the above-mentioned points, the hierarchical analysis model is constructed as shown in Figure 2.

The basic level of the model: decision target refers to the final derived result; criterion layer is the criteria for the model judgment to make a decision; program layer refers to each specific program limited by the decision target and criterion layer. In the model, the highest risk factor is used as the target: severity and incidence as the criterion; four types of risk: sports instruction, partner cooperation, personal factors, and sports combination as the alternative. Next, a comparison matrix is constructed and solved, and finally the highest risk category is determined in a logical way, and those risk exposures with higher incidence and more severe consequences are identified and focused on [21–25].

The relative importance of the above-given four factors was compared between the two under the constraints of the criterion level. The importance ratings of coaches and athletes on the seven major exposures of the four risk categories were first arithmetically averaged in terms of categories and then weighted in terms of the ratio of the number of coaches and athletes participating in the study to obtain the final values of the matrix factors, and the judgment matrix was constructed.

The fourth-order matrix *A* formed is as follows (*A*_*ij*_ is the ratio of importance between risks *ij*, *A*_*ji*_=1/*A*_*ij*_):

(1) $$\begin{array}{c} A=\left[\begin{array}{cccc} 1.00 & 4.00 & 7.00 & 9.00\\ 0.25 & 1.00 & 4.00 & 6.00\\ 0.14 & 0.25 & 1.00 & 3.00\\ 0.11 & 0.16 & 0.33 & 1.00 \end{array}\right]. \end{array}$$

To achieve the sports training injury risk assessment model, the big data fusion scheduling method is used for big data information sampling of sports training injury risk assessment, combined with the statistical information mining method for sports training injury risk assessment, dividing the level of sports training injury risk assessment *X*^(0)^, into *N* levels, as *X*^(1)^, *X*^(2)^,…, *X*^(*N*)^ , i.e. *X*^(0)^=∪_*i*=1_^*N*^*X*^(*i*)^ , with fuzzy feature distributed mining method for statistical analysis and optimal assessment of sports training injury risk, establishing a big data analysis model for sports training injury risk assessment, adaptive learning for sports training injury risk assessment, and obtaining a statistical function for sports training injury risk assessment as.

The above-given equation is a big data fusion model of sports training injury risk assessment for quantitative analysis of sports training injury risk assessment [26, 27], and the correlation distribution relationship of the constraint covariate set *R*^*N*^, *X*^*N*^ of sports training injury risk assessment is established as follows.

Combining the autocorrelation feature matching method for sports training injury risk assessment big data sampling, according to the sampling results for sports training injury risk optimization evaluation and decision making. The feature matching function of sports training injury risk is established, {*x*(*t*_0_+*i*Δ*t*)},  *i*=0,1,…, *N* − 1. The optimization-seeking trajectory of machine learning is as follows.

The fuzzy parametric identification of sports training injury risk assessment is carried out by using output stability gain assessment and the fuzzy decision method is constructed as follows.

In the following equation, *λ* represents the fuzzy distribution factor of the big data for sports training injury risk assessment, combined with the statistical feature analysis method for sports training risk assessment. The sports training injury risk assessment is obtained as follows:

(2) $$\begin{array}{c} \sum_{s_{c}\in S^{2}}p\left\{C_{k}^{l}/A_{k}^{i}B_{k}^{b}\right\}p\left\{A_{k+1}^{j}/A_{k}^{i}B_{k}^{b}C_{k}^{l}\right\} \end{array}$$

The linear fit equation for the risk assessment of physical training injuries is

(3) $$\begin{array}{c} p_{\text{id}}^{\text{new}}=\left\{\begin{array}{cc} p_{\text{id}}+m\left(\;\right)\left(X_{\text{max}}-p_{\text{id}}\right) & \text{ if }m\left(\;\right)>0\\ p_{\text{id}}+m\left(\;\right)\left(p_{\text{id}}-X_{\text{min}}\right) & \text{ if }m\left(\;\right)\leq 0 \end{array}\right). \end{array}$$

The similarity analysis method is used for adaptive assessment of sports training injury risk, and the fuzzy control in the process of sports training injury risk assessment is as follows:

(4) $$\begin{array}{c} SL_{i}=\left\{\begin{array}{cc} L_{i} & \text{if }i=1\\ N_{ew} & \text{otherwise} \end{array}.\right) \end{array}$$

The association rule distribution function for sports training injury risk assessment is *M*_*h*_ , and the joint association rule mining method is used to obtain a finite dataset of association dimensional distribution for sports training injury risk assessment.

(5) $$\begin{array}{c} X=\left\{x_{1},x_{2},\ldots ,x_{n}\right\}\subset R^{2} \end{array}$$

Among them, the sports training injury risk assessment contains *n* samples, and the expert system analysis model of sports training injury risk assessment is established, and the control sample function is obtained as *x*_*i*_, *i*=1,2,…, *n*, and the feature quantity of sports training injury risk assessment is obtained by combining the hierarchical gray-scale correlation analysis method *p*_*q*_, and the quantitative relationship of sports training injury risk assessment is as follows.

To sum up, the analysis, to achieve the optimization of sports training injury risk and improve sports training injury risk control.

## 4. Overall Design of the Artificial Intelligence Web-Based Teaching Platform

### 4.1. Overall Design of the Web-Based Teaching Platform

The Artificial Intelligence Network Teaching Platform, with its efficient, remote, and resource-sharing features, allows advanced and rich course resources to be shared on the Internet, enabling teachers and students to download and share electronic resources such as teaching contents and cases, microlessons and courseware, and scientific research results and papers. Students can rely on the flipped classroom teaching model in the online learning space to customize and personalize their learning or rely on the teaching platform for interactive and shared communication and as a supplementary teaching tool to traditional teaching.

### 4.2. Design of the Database

To design an effective database, a systems engineering perspective is required. As the website is an AI web-based teaching platform, it has a wide range of course resources and therefore a large number of corresponding data sheets, including article system Data Sheet; Downloading system Data Sheet; Electronic lesson plans Data Sheet; FLASH System Data Sheet; Classified information Sheet; Electronic lesson plans Data Sheet. The electronic lesson plans Data Sheet; the FLASH System Data Sheet; the Classified information Sheet; the Photo System Data Sheet, etc. The electronic lesson plans and FLASH System Data Sheet are shown in Tables 1 and 2.

#### 4.2.1. Electronic Lesson Plan Data Sheet

The Electronic lesson plans Data Sheet is an information management tool for electronic lesson plans, which includes: title, special attributes, title image, and release time information. The corresponding fields are shown in Table 1.

#### 4.2.2. FLASH System Data Sheet

The FLASH System Data Sheet is the information management for FLASH files, including Title, Special Attributes, Author, FLASH Address, FLASH Width, and FLASH Height. The corresponding fields are shown in Table 2.

## 5. Functional Implementation of a Web-Based Platform for Artificial Intelligence Courses

### 5.1. Experiments

Pareto analysis was applied to assess the overall risk factors of sports training, and the results of the overall risk assessment of sports training were obtained, as shown in Table 3.

The artificial intelligence course network teaching platform is divided into the following six functional modules:

  Course introduction: provide users with course introduction and courseware materials.
  Teaching team: briefly introduce the teaching team of the course website, so that users can have a certain understanding of the teachers of the website.
  Teaching achievements: the teaching achievements module is a platform for teachers' achievements display and sharing. Users can browse teachers' teaching achievements on the website, such as teachers' papers, certificates, and projects.
  Teaching resources: including teaching resources such as course content based on flipped teaching concepts (WeChat, PPT, WeChat platform, etc.), course cases, and syllabus based on task-driven teaching mode. Users can freely choose the required materials for browsing and learning.
  Learning garden: the learning garden is a display platform for scientific papers and excellent homework and a platform for interactive communication between teachers and students, providing users with reference materials for learning and reference.
  Data download: it mainly completes the function of uploading and downloading electronic resources. The courseware includes relevant videos, a question bank, and courseware.

### 5.2. Platform Implementation

According to the function of the platform, it realizes six modules: course introduction, teaching team, teaching results, teaching resources, learning garden, and data download. Different modules correspond to different pages, with simple structure and clear content. The function menu of the website is expanded in the form of a single row list, which makes the whole page appear orderly, concise, and clear. Users can easily browse the content of the website according to their needs and introduce the implementation process of the platform with the login interface and teaching resource module of the website.

#### 5.2.1. Login Operation

This module is the system login interface. Its function is to detect whether the login user is legal and prevent illegal users from invading the system by verifying their user name and password. The system shall automatically judge the correctness of the user name and password entered. If the login is normal, the system shall record the current user name so that other operations can be assigned with appropriate permissions. The system login interface and website home page are shown in Figures 3 and 4.

#### 5.2.2. Teaching Resource Module

The teacher resource module is the main functional module of the course platform. The module includes: teaching cases, teaching content, teaching video, teaching calendar, microclass, and PPT. Administrators release teachers' teaching videos and other teaching content to provide users with browsing and learning resources. After users select the required course resources and download them, they can view the course resources such as the course content and teaching cases [21, 22].

*(1) Course Content Module*. In the course content module, the teaching platform integrates the microcourse and diagnosis and treatment system of flipped classroom concept [23]. The flipped classroom is a new teaching model, which is composed of three basic elements: technical elements (mainly microvideo), process elements (before class-in class-after class), and environmental elements (intelligent diagnosis learning system). Flipped classroom focuses on the whole process of teaching activities, focuses on the teaching interactive behavior of teachers and students supported by a multimedia environment, and focuses on the active awakening of students' innovative spirit [24]. Based on this new concept of “flipped classroom,” this paper designs the teaching design process and mode based on the public platform, as well as how to carry out the learning and interactive process of the micromobile course based on the WeChat public platform and develops the microcourse of principles of artificial intelligence based on the WeChat public platform and the corn pest diagnosis and treatment system in smart agriculture, as shown in Figures 5 and 6.

Figure 5 shows the characteristics of the flipped classroom. Teachers and students use multimedia technology to interact and communicate in time in the classroom. This teaching method plays a very good role in cultivating students' autonomous learning ability, autonomous problem discovery, and problem-solving ability.  Figure 6 is the interface of the grass damage diagnosis and treatment system. The system is the application of artificial intelligence in grass damage diagnosis and treatment. Students can learn independently after class and diagnose grass damage by themselves [25–27].

## 6. Effectiveness of Aesthetic Informatics

Campus culture has a subtle effect on teachers and students, influencing both their values and the learning atmosphere on campus. An information-based campus environment can enhance the breadth and depth of campus culture communication, break the constraints of time and space, enhance the attractiveness of campus culture, stimulate students' curiosity and creativity, and improve the efficiency of campus culture construction. Firstly, schools should actively use information technology to promote communication between students and the outside world and to stimulate their imagination and creativity in beauty. As shown in Figure 7 for its 3D distribution of resource use, schools use the network to share campus aesthetic culture resources, which can create a campus culture building platform for teachers, students, and parents to participate in, bringing individual campus culture in line with popular culture. Schools should use new media technology to create an information-based aesthetic environment for students, such as providing them with brightly colored pictures, pleasant music, lively animations, and virtual simulation images so that they can perceive the charm of campus aesthetic culture in many ways.

Schools should train teachers in all subjects at the generalist level of aesthetic education, set out beauty design requirements for teaching design and courseware, regulate teachers' teaching language and processes in terms of beauty, and integrate aesthetic education organically into the teaching of all subjects. As shown in the radar diagram of the functions of different resources in schools in Figure 8, the practice of specialized courses in aesthetic education should be increased so that students can perceive first-hand what is around them. Schools can also try to integrate humanistic customs and local characteristics of landscape resources from around the world; for example, by offering a weekly practical lesson on aesthetic education and allowing teachers to take students outside for viewing and learning. Such a teaching approach that combines aesthetic education with local natural and humanistic landscapes can broaden the scope of aesthetic education, allowing students to appreciate the beauty of their hometowns and lives while enriching their own aesthetic world and enhancing their own aesthetic sensibilities.

Exploring information technology to facilitate cooperation between home, school, and society Aesthetic education in the new era requires schools to co-ordinate and integrate social resources to implement the goal of enhancing students' aesthetic abilities in a home-school approach. With the increasing improvement of the school's information technology hardware construction and the increasing awareness of information technology, the learning effect of different campus websites, as shown in Figure 9, which can release school information or communicate with parents and society. Schools should pay full attention to and make use of the social resources around them, using information technology as a medium to design feasible aesthetic education collaborative projects to benefit students.

## 7. Conclusions

In the process of promoting aesthetic education, as the main body, the school has many shortcomings. Schools should strive to find strong and feasible initiatives in terms of system construction, teaching methods, teachers, digital resources, and improvement of conditions to find a breakthrough and anchor point for information-based aesthetic education and enhance students' aesthetic literacy. This paper combines the teaching objectives of the AI course and the characteristics and steps of the task-driven teaching method to develop an online teaching platform for the core AI course, which breaks the time and space limitations of the traditional teaching mode and enables teachers and students to learn and communicate anytime and anywhere, rather than being confined to the classroom. This provides a new mode of learning for the core AI course and has a positive effect on students' learning [19].

## Figures and Tables

**Figure 1:** Flow chart of a traditional genetic algorithm.

**Figure 2:** Hierarchical decision model for high-risk factors.

**Figure 3:** System login interface.

**Figure 4:** Website home page.

**Figure 5:** Interaction process of micro class.

**Figure 6:** Grass damage diagnosis and treatment system.

**Figure 7:** Utilisation of learning resources.

**Figure 8:** Radar chart of school resources and student status.

**Figure 9:** School teaching platform conversion matrix.

**Table 1:** Electronic lesson plan datasheet.

Field name	Field identification	Field type
Title	Title	System field
Specialfield	Special properties	System field
Titlepic	Title picture	System field
Newstime	Release time	System field

**Table 2:** Fash system datasheet.

Field name	Field identification	Field type
Title	Title	System field
Specialfield	Special properties	System field
Newstime	Release time	System field
Titlepic	Title picture	System field
Flashwriter	Author	VARCHAR (30)
E-mail	Author e-mail	VARCHAR (80)
Star	Work level	TIV NYINT(1)
Filesize	File size	VARCHAR (16)
Flashurl	Flash address	VARCHAR (255)
Width	Flash width	VARCHAR (12)
Height	Flash height	VARCHAR (12)
Flashsay	Introduction to works	Text

**Table 3:** Sports training risk factors category statistics.

No.	Risk factor category	Frequency	Cumulative percentage (%)
A-a	Student movement behavior risk	162	20.12
C-b	Sports equipment risk	148	39.69
C-a	Activity venue risk	139	55.36
A-b	Student self-management risk	125	71.03
B-a	School safety management risk	100	82.55
D-b	Man-made environment risk	75	92.36
B-b	School medical supervision risk	35	96.77
D-a	Natural environment risk	28	100

## Data Availability

The experimental data used to support the findings of this study are available from the corresponding author upon request.

## References

[1] Pan Y., Zhang L. (2021). Roles of artificial intelligence in construction engineering and management: a critical review and future trends. *Automation in Construction*.

[2] Kong F. (2020). Application of artificial intelligence in modern art teaching. *International Journal of Emerging Technologies in Learning (iJET)*.

[3] Xie X., Pan X., Shao F., Zhang W., An J (2022). MCI-Net: multi-scale context integrated network for liver CT image segmentation. *Computers & Electrical Engineering*.

[4] Abiodun O. I., Jantan A., Omolara A. E., Dada K. V., Mohamed N. A., Arshad H. (2018). State-of-the-art in artificial neural network applications: a survey. *Heliyon*.

[5] Sil R., Roy A., Bhushan B., Mazumdar A. K. Artificial intelligence and machine learning based legal application: the state-of-the-art and future research trends.

[6] Yigitcanlar T., Desouza K. C., Butler L., Roozkhosh F. (2020). Contributions and risks of artificial intelligence (AI) in building smarter cities: insights from a systematic review of the literature. *Energies*.

[7] Lu Y. (2019). Artificial intelligence: a survey on evolution, models, applications and future trends. *Journal of Management Analytics*.

[8] Tao X. I. E., Zhang C., Xu Y. (2021). Collaborative parameter update based on average variance reduction of historical gradients. *Journal of Electronics and Information Technology*.

[9] Zhengwan Z. H. A. N. G., Chunjiong Z. H. A. N. G., Hongbing L. I., Tao X. I. E. (2020). Multipath transmission selection algorithm based on immune connectivity model. *Journal of Computer Applications*.

[10] Mosavi A., Varkonyi-Koczy A. R. (2017). *Integration of machine learning and optimization for robot learning*.

[11] Ahmad T., Zhang D., Huang C. (2021). Artificial intelligence in sustainable energy industry: status Quo, challenges and opportunities. *Journal of Cleaner Production*.

[12] Gupta A., Ong Y. S., Feng L. (2018). Insights on transfer optimization: because experience is the best teacher. *IEEE Transactions on Emerging Topics in Computational Intelligence*.

[13] Salehi H., Burgueño R. (2018). Emerging artificial intelligence methods in structural engineering. *Engineering Structures*.

[14] Auerbach J. E., Concordel A., Kornatowski P. M., Floreano D. (2019). Inquiry-based learning with robogen: an open-source software and hardware platform for robotics and artificial intelligence. *IEEE Transactions on Learning Technologies*.

[15] Yoon D. M., Kim K. J. (2015). Challenges and opportunities in game artificial intelligence education using angry birds. *IEEE Access*.

[16] Yang X., Wang Y., Byrne R., Schneider G., Yang S. (2019). Concepts of artificial intelligence for computer-assisted drug discovery. *Chemical Reviews*.

[17] Xie X., Pan X., Zhang W., An J. (2022). A context hierarchical integrated network for medical image segmentation. *Computers & Electrical Engineering*.

[18] Sejnowski T. J. (2020). The unreasonable effectiveness of deep learning in artificial intelligence. *Proceedings of the National Academy of Sciences*.

[19] Fahle S., Prinz C., Kuhlenkötter B. (2020). Systematic review on machine learning (ML) methods for manufacturing processes–Identifying artificial intelligence (AI) methods for field application. *Procedia CIRP*.

[20] An P., Wang Z., Zhang C. (2022). Ensemble unsupervised autoencoders and Gaussian mixture model for cyberattack detection. *Information Processing & Management*.

[21] Liu B. (2019). BioSeq-Analysis: a platform for DNA, RNA and protein sequence analysis based on machine learning approaches. *Briefings in Bioinformatics*.

[22] Wu M., Payshanbiev A., Zhao Q., Yang W. (2021). Nonlinear optimization generating the tomb mural blocks by GANS. *Applied Mathematics and Nonlinear Sciences*.

[23] Lin X., Wu J., Mumtaz S., Garg S., Li J., Guizani M. (2021). Blockchain-based on-demand computing resource trading in IoV-assisted smart city. *IEEE Transactions on Emerging Topics in Computing*.

[24] Li J., Zhou Z., Wu J. (2019). Decentralized on-demand energy supply for blockchain in Internet of things: a microgrids approach. *IEEE Transactions on Computational Social Systems*.

[25] Duan W., Gu J., Wen M., Zhang G., Ji Y., Mumtaz S. Emerging technologies for 5G-IoV networks: applications, trends and opportunities. *IEEE Network*.

[26] Jiang D., Wang F., Lv Z. (2021). QoE-aware efficient content distribution scheme for satellite-terrestrial networks. *IEEE Transactions on Mobile Computing*.

[27] Mocanu E., Mocanu D. C., Nguyen P. H. (2019). On-line building energy optimization using deep reinforcement learning. *IEEE Transactions on Smart Grid*.

